This article has been retracted.

# Impact of drying methods on composition and functional properties of date powder procured from different cultivars

**DOI:** 10.1002/fsn3.1081

**Published:** 2019-06-04

**Authors:** Nighat Raza, Muhammad U. Arshad, Faqir M. Anjum, Farhan Saeed, Abid A. Maan, Huma Bader Ul Ain

**Affiliations:** ^1^ Institute of Home and Food Sciences Government College University Faisalabad Punjab Pakistan; ^2^ The University of Gambia Gambia Gambia; ^3^ National Institute of Food Science & Technology University of Agriculture Faisalabad Pakistan

**Keywords:** date pit powder, nutritional attributes, oven drying, physicochemical properties, spray drying

## Abstract

The present study was designed to evaluate the effect of two different drying methods, that is, spray drying and oven drying on physicochemical and nutritional attributes of date flesh powder of dhakki, aseel, and rabi varieties. Date powders were prepared using mixture of maltodextrin and acacia gum (50:50) as drying aid at the rate of 0.4 kg per 1.0 kg of date fruits (dry weight basis). The oven‐drying conditions were 60°C for 48 hr, whereas in spray drying, flow rate of 30 ml/min at 150°C was maintained. Date powder was obtained in both treatments from three varieties. Nutritional profile in all six powders was explored specifically with quantification of sugars using HPLC‐RI, followed by physicochemical characterization. The total phenolic compounds, color (L*a*b* values), hygroscopicity, bulk density, wettability, solubility index, and glass transition temperatures (using differential scanning calorimetry, DSC), were determined for the date powders. The nutritional profile and total phenolic contents and sugars (sucrose, fructose, and glucose) were significantly different for the varieties, while treatments showed insignificant effect. The physicochemical characteristics of date powder varied significantly with respect to the date varieties. The colored values were affected due to treatments also, and the spray‐dried powders showed better color values. The drying methods also showed effects in some parameters such as wettability time. Similarly, bulk density was different in both treatments for rabi and aseel. The glass transition temperatures were significantly varied in varieties due to difference in sugar contents, but within the treatments, they remain unaffected. The highest glass transition temperature of spray‐dried rabi was 53.2 ± 1.31°C.

## 1 INTRODUCTION

Drying is designated as a powerful processing technique to preserve food materials. A number of diversified techniques are currently in practice for drying of solutions and whole food materials in solid states, pastes, and sheets, hence providing broad spectra among all food preservation process (Jaya, Das, & Mani, 2006). The drying of commodity and conversion into complete powder using a raw‐material‐specific technique is very common nowadays. Milk and egg powders are very common examples. Fruits powders are also getting popularity due to ease of preservation, handling, transport, and safe storage (Phisut, 2012).

The major problem encountered by the food processors in processing is stickiness owing to the higher sugar contents of fruits (Jaya et al., 2006). These low molecular weight sugars and number of organic acids are very hygroscopic in powdered form and therefore hampered during drying, processing, and proper storage. In food industry, drying aids (anticaking agents) are used to deal with such situations (Yousefi, Emam‐Djomeh, & Mousevi, 2011). In the production of tamarind powder, the maltodextrin at various levels (0%–15%) was used with temperature ranged from 55 to 70°C, which results in better texture of the powder with higher maltodextrin percentage (Ekpong, Phomkong, & Onsaard, 2016). The concentration of maltodextrin was also optimized along with variable spray‐drying condition for the production of guava powder that resulted in significantly different products due to different conditions (Patil, Chauhan, & Singh, 2014). Other drying aids can be used depending upon the end user, such as maltodextrin of different DE, acacia gum, and isolated proteins can be added in the fruit pulps before applying drying techniques in order to minimize stickiness in the final product (Caparino et al., 2012; Ferrari, Germer, Alvim, & Mauricio de Aguirre, 2013; Patil et al., 2014; Phisut, 2012). Likewise, the application of acacia gum was compared with the maltodextrin in an experiment that proved it better than maltodextrin and gave maximum production of apricot fruit (Razzaq et al., 2017). Acacia gum as carrier agent not only provide anticaking properties but also act as a source of high‐quality soluble fiber that could be used by intestinal microflora as prebiotic and provide extra benefits beyond basic nutrition and processing tool (Cherbut, Michel, Raison, Kravtchenko, & Severine, 2003). Therefore, addition of acacia gum equipped the final product with nutraceutical properties.

Date fruit is labeled as energy‐dense food with almost all essential micronutrients, more than 15 minerals, and enriched with vitamins (Al‐Farsi & Lee, 2008). Pakistan is 7th largest exporter of the date fruit. The energy density of date fruit is 314 kcal/100 g of date flesh, and it provides almost all essential nutrients (Al‐Shahib & Marshall, 2003) comprised of fructose and glucose when we consider the macronutrients while micronutrient contribution of dates is also worth considering. It is an established fact that date fruit possess different nutraceutical properties due to the presence of significant amount of dietary fiber, vitamins, carotenoids, phenolics, and antioxidants. These groups have been proved to provide different health benefits such as nephroprotection, neuroprotection, and hepatoprotection. It may also show anticarcinogenic, antihyperlipidemic, and anti‐inflammatory properties (Chandrasekaran & Bahkali, 2013; Dayem et al., 2016; Khalid, Khalid, Khan, Ahmed, & Ahmad, 2017).

The premium quality dates are mostly consumed freshly. But in country such as Pakistan where postharvest loses are more than 40%, excess produce should be handled the way it does not get wasted (GOP, 2016). High moisture contents can increase the onset of degeneration and increase the perishability of the dates; therefore, drying is indispensable in order to enhance the shelf life of the dates (Falade & Abbo, 2007). Many attempts have been made earlier to process the dates in the form of date jam, date syrups, date chutneys, and date bars. The present study is an attempt to produce a free‐flowing powder from the date flesh using two different drying techniques (Sablani, Shresta, & Bhandari, 2008). Three commercially available date varieties were collected and put for spray drying and oven drying using a blend of anticaking agents in ratio of 1:1, and then, the resultant products were tested for their nutritional and physicochemical properties. This was a novel approach to use two carriers simultaneously in the same proportion as a drying aid in order to develop a nutraceutical date powder.

## 2 MATERIALS AND METHODS

### 2.1 Procurement of raw material

Three commercially available date varieties (aseel, rabi, and dhakki) were collected from Date Palm Research Institute, Jhang, Punjab, Pakistan. Analytical grade chemicals were purchased from Merck, Oxide, and Applichem.

### 2.2 Preparation of date powders

The date varieties procured were subjected to initial treatment for removal of inedible part and any adhered foreign particle, that is, washing, depitting, and steaming. These samples were subjected to drying treatments.

#### 2.2.1 Carrier agent

For preparation of free‐flowing powder, a combination of acacia gum and maltodextrin was used as carrier agents in order to reduce the stickiness in resultant product, because they are highly heat‐stable.

### 2.3 Oven drying

Depitted and steamed dates were blended with carrier agent (maltodextrin and gum Arabic 1:1) in a blender (Kenwood AT358 Thermoresist™) to get their paste. The paste was spread in plate evenly in the form of thin sheet and subjected to oven drying at 60°C for 24 hr. After 24 hr, dried sheets were placed in a grinding mill. After grinding, a free‐flowing powder was obtained that was immediately stored into the airtight jars for further analyses (Sablani et al., 2008).

### 2.4 Spray drying

The dates were grounded in a blender with water and drying aids in the same concentration used in oven‐drying method. Prepared date paste was diluted with water in ratio of 20:80 to make slurry. During final feedstock preparation, the slurry was sieved through an 80‐mesh sieve to avoid any blockage in the nozzle. The conditions of pilot‐scale spray drier (Anhydro) was kept constant at temperature 150°C and flow rate 30 ml/min. The resultant free‐flowing powder was stored in ziplock polyethylene bags immediately (Manickavasagan et al., 2015).

### 2.5 Analyses of date powders

#### 2.5.1 Proximate analysis

The moisture contents, crude fat, crude proteins, crude fiber, and ash contents were determined by standard methods (AOAC, 2012).

### 2.6 Sugar analysis

#### 2.6.1 Quantification of mono/disaccharides

The quantification of monosaccharides (fructose and glucose) and disaccharide (sucrose) was done through high‐performance liquid chromatography (HPLC) using RI (refractive index) detector according to the method of Karkacier, Erbas, Uslu, and Aksu (2003) with some modifications.

### 2.7 Extraction

The 10 g powder sample was homogenized along with 40 ml of methanol at a magnetic stirrer at 300 rpm, supernatant was increased by adding 50 ml methanol, and this extract was reduced in the volume by rotary vacuum evaporator. The concentrated solution was filtered through filter paper and was stored in plastic bottles at 4°C until analyzed. The extraction from each variety was done in triplicate.

### 2.8 Chromatographic system

High‐performance liquid chromatography system from Agilent 1100 series was used with reverse‐phase C18 column in octadecyl sulfonate packing, with length 25 cm, diameter 2.5 mm, and pore size of 5 micron. Mobile phase was acetonitrile: water in the ratio of 75:25. Flow rate was 0.9 ml/min with isocratic elution with refractive index detection. Procured standards and extracted samples were introduced in the system through PVDF 0.45‐µm syringe. The retention time for each standard and sample was 30 min approximately, as the whole process was controlled and connected to computer software to directly quantify the sugars.

### 2.9 Total phenolic contents

Analysis of total phenols was carried out by Folin–Ciocalteu reagent calorimetrically (Blainski, Cristiny, & Palazzo, 2013).

### 2.10 Procurement of standard

Gallic acid was procured from Sigma‐Aldrich. Standards were prepared in water (50, 100, 150, and 200 mg) to establish a calibration curve.

### 2.11 Extraction and estimation of TPC

Ten gram of powder sample was taken in 90 ml of (99%) methanol and stirred for half an hour on magnetic stirrer and filtered through Whatman No. 41 paper to get the supernatant, and the residue was washed three times, concentrated in a vacuum dryer, and stored below 20°C until analyzed. 0.125 ml of the extract was taken in a conical flask, and 1.8 ml Folin–Ciocalteu reagent was added. Dilution was done (10×) by adding water and kept for 6 min at room temperature. The reaction mixture was loaded with 1.2 ml of sodium carbonate (15%) and kept for 90 min at 25°C. The absorbance was measured at 765 nm, and results were expressed as milligram of gallic acid equivalents/gram powder weight.

### 2.12 Physicochemical properties of date powders

#### 2.12.1 Color

The color of spray‐dried date powders was determined using a color flex meter (Hunter Association laboratory, Inc.) with CIELAB (L*, a*, and b*) (10° observer at D65 illuminant). The illumination chamber diameter was 25.4 mm. The instrument was calibrated with black and white standard tiles before each experiment. The results were expressed as Hunter color values of “L*,” “a*,” and “b*,” where the “L*” value is used to denote lightness (+) and darkness (−), the “a*” value is used to denote redness (+) and greenness (−), and the “b*” value is used to denote yellowness (+) and blueness (−).

#### 2.12.2 Bulk density

The bulk density of powders was determined as mass per unit of volume (WHO, 2012) and was expressed as g/cm^3^.

#### 2.12.3 Wettability time

The wettability time was measured by IDF method No. A5b revised in 2009 (GEA, 2009). In brief, 10 g sample was weighed in a petri plate and 250 ml water was taken in a beaker. A glass plate was placed on the beaker where sample was placed. The whole sample was introduced to water surface in 2.5 s. The time was noted from touching of powder to the surface of water till all the particles became wet and denoted as wettability time.

#### 2.12.4 Water activity

Water activity was measured by a precalibrated bench‐top water activity meter (Model: Aqua Lab 4TE, Decagon Devices, Inc.) at 30°C ± 1.

#### 2.12.5 Solubility index

One gram of sample from each type of powder was added to 100 ml of distilled water. Mixing was done on a magnetic stirrer, and after complete mixing, it was allowed to stand at 37°C for 30 min. The solution (dispersed date powder) was subjected to centrifugation (3,000 *g* for 5 min). A 25 ml aliquot from the supernatant was dried at 105°C until constant weight in a hot air oven. The solubility index (%) was calculated by taking the weight difference (Caparino et al., 2012).

#### 2.12.6 Hygroscopicity

One gram powder sample with water activity <0.02 sample was taken and spread on petri plates evenly to ensure high surface area. Petri plate was placed in a desiccator with higher relative humidity, that is, 76%. The weight gain was noted after every 2 hr in 24 hr till a constant weight that showed capacity of the powder to carry highest amount of the moisture from the atmosphere. Weight gain was expressed as gram of water/gram of powder (Manickavasagan et al., 2015).

#### 2.12.7 Glass transition temperatures

Glass transition temperature (*T*_g_) of date powders with water activity below 0.2 was measured using differential scanning calorimeter (DSC, Q2000, TA Instruments), following the procedure described by Syamaladevi, Sablani, Tang, Powers, and Swanson (2008). The calorimeter was calibrated for heat flow and temperature using standard indium and sapphire. Twelve to sixteen milligrams of each date powder sample was sealed in an aluminum pan (volume of 30 L), cooled down from 25 to −90°C using liquid nitrogen, and equilibrated for 10 min. The samples at −90°C were scanned to 90°C, then cooled down to 25°C. Scanning of all samples was carried out using the same heating and cooling rate of 5°C/min. To avoid condensation on the surface of the powder particles, a nitrogen carrier gas was purged at a flow rate of 50 ml/min in the aluminum pan. The inception (*T*_gi_), mid (*T*_gm_), and end point (*T*_ge_) values of the date powders were determined by finding the vertical shift in the heat flow–temperature diagram. All measurements were performed in duplicate.

## 3 RESULT AND DISCUSSION

### 3.1 Proximate analysis

Proximate profiling (Table 1) indicated that moisture contents ranged from 2.53 ± 0.12% to 1.47 ± 0.05% for spray‐dried dhakki and oven‐dried rabi, respectively. Dates as pronounced source of minerals ensued in higher ash contents in all cultivars therefore showed nonsignificant difference for cultivars. Treatments showed insufficient effect on drying. Among three, only dhakki showed slightly higher contents that were 5.76 ± 0.29% and 5.71 ± 0.09% in oven‐dried and spray‐dried dhakki, respectively. The comparison of all varieties for protein level revealed that both dhakki and aseel possessed almost equal levels of proteins, while rabi with slightly higher level with values 5.61 ± 0.19% and 4.99 ± 0.29% for drying treatments. So, the protein contents differed significantly among varieties, while drying methods have no significant difference according to the findings. It has been reported earlier that dates contain very little amount of crude fat (<1%) (Gallo, Llabot, Allemandi, Bucala, & Pina, 2011). Fat contents in all three varieties were varied quite significantly, but there was no significant difference among treatments. Crude fiber contents remained unaffected during the treatments, whereas they varied among varieties. The crude fiber contents were higher in dhakki with values 8.66 ± 0.27% and 7.90 ± 0.21% for spray‐dried and oven‐dried dhakki, respectively. The NFE contents varied among the varieties to lesser extent, whereas drying treatments revealed nonsignificant difference.

**Table 1:** Means ± *SD* for proximate composition (%) of date powders

Variety	Treatment	Moisture	Crude protein	Crude fat	Crude fiber	Ash	NFE
Rabi	OD	1.55 ± 0.09^c^	5.61 ± 0.19^a^	0.87 ± 0.06^a^	6.46 ± 0.2^c^	4.73 ± 0.18^d^	80.64 ± 0.36^a^
	SD	1.47 ± 0.05^c^	4.99 ± 0.29^ab^	0.86 ± 0.11^a^	6.63 ± 0.18^c^	5.62 ± 0.26^abc^	80.71 ± 0.57^a^
Aseel	OD	2.39 ± 0.15^ab^	4.57 ± 0.42^bc^	0.34 ± 0.06^c^	7.73 ± 0.51^b^	5.18 ± 0.25^cd^	79.06 ± 0.42^b^
	SD	2.35 ± 0.2^ab^	4.70 ± 0.50^bc^	0.33 ± 0.08^c^	7.67 ± 0.08^b^	5.28 ± 0.32^bc^	80.28 ± 0.87^a^
Dhakki	OD	2.53 ± 0.12^a^	4.1 ± 0.38^c^	0.67 ± 0.05^b^	7.67 ± 0.21^b^	5.76 ± 0.29^a^	79.1 ± 0.32^b^
	SD	2.28 ± 0.15^b^	4.57 ± 0.27^bc^	0.73 ± 0.03^b^	8.72 ± 0.27^a^	5.71 ± 0.09^ab^	78.45 ± 0.51^c^

Note

Means carrying different letters are significantly different (*p* < 0.05).

### 3.2 Monosaccharide/disaccharide quantification

The analysis revealed that there were only two dominant types of sugars, fructose and glucose, while sucrose was present in lesser quantity. For glucose, there was nonsignificant difference (*p* > 0.05) within the treatments, while varieties showed significant difference (Table 2). Among varieties, rabi depicted higher contents of glucose ranged from 32.55 ± 0.15 to 32.43 ± 0.65 in both treatments, compared to aseel and dhakki where it ranged from 26.95 ± 0.69 to 28.5 ± 0.46 for oven drying. Fructose contents were higher in aseel (33.51 ± 0.6 for oven dried, 33.75 ± 0.32 for spray dried) as compared to rabi and dhakki. Drying treatment showed negligible effect on sugar contents but varied significantly among the varieties. Owing to such high contents of invert sugars and presence of acacia gum (known for abating the hyperglycemia), date powder was used as low‐glycemic tabletop sweetener for diabetic patients.

**Table 2:** Means for different sugars (G/100 g) of date powders

Variety	Treatment	Sucrose	Glucose	Fructose
Rabi	OD	2.67 ± 0.48^a^	32.55 ± 0.15^a^	30.29 ± 0.4^b^
	SD	2.63 ± 0.31^a^	32.43 ± 0.65^a^	30.96 ± 0.55^b^
Aseel	OD	2.09 ± 0.13^a^	26.02 ± 0.69^d^	33.51 ± 0.6^a^
	SD	2.56 ± 0.14^a^	26.95 ± 0.56^cd^	33.75 ± 0.32^a^
Dhakki	OD	2.38 ± 0.48^a^	28.5 ± 0.83^b^	31.34 ± 0.57^b^
	SD	2.59 ± 0.28^a^	27.13 ± 0.06^bc^	32.18 ± 0.2^b^

Note

Means carrying different letters are significantly different (*p* < 0.05).

### 3.3 Total phenolic contents of date powders

Higher TPCs were found in oven‐dried dhakki 438.94 mg/100 g followed by spray‐dried dhakki, that is, 411.77 mg/100 g (Figure 1). The lower contents were found in aseel, that is, 76.92 and 77.24 mg/100 g for spray‐dried and oven‐dried aseel, respectively. Despite the varieties, the oven‐dried powders showed slightly higher concentration of phenolics as compared to spray‐dried powders. Phenolic contents of date variety are symbol of its nutraceutical properties owing to the antioxidant potential (Baliga, Baliga, Kandathil, Bhat, & Vayalil, 2011; Khalid et al., 2017).

**Figure 1:** Means of total phenolic content (mg/100 g) of date powders

### 3.4 Physicochemical properties of date powders

#### 3.4.1 Color

The higher value of “L*” among all varieties was observed from spray‐dried aseel followed by oven‐dried aseel, and the difference among the varieties was quite significant because actual color of varieties was different. Rabi was darker compared to aseel and dhakki. The drying technique also affected the “L*” value of the powders, and in all three varieties, spray‐dried varieties possessed slightly higher values referred to the lighter color, while oven dried with low *L* values denoted to the darker colors. Dhakki with higher “a*” value 4.24 ± 0.11 showed the redness, and the “L*” pattern repeated itself and showed that both treatments produced powders with different “a*” values (Table 3), wherein color degradation was greatly influenced by high processing temperatures and the time period. The dark color in oven‐dried date powder was due to Maillard reaction, chemical reactions between sugars and proteins (Potter & Hotchkiss, 1995). Moreover, caramelization of sugars in dates occurred due to long exposure of temperature causative to darkening during drying. The already dominant color of date paste was brown, and the hunter color b* (yellowness) was represented to elaborate the color difference in the resulted date powders affected by drying process in the distinguished variety. Nonsignificant difference was observed in b* value (yellowness) between oven‐ and spray‐dried date powders, while a significant difference between varieties was noticed (*p* ˃ 0.05). Although dhakki and aseel did not show that much difference, the difference from rabi was highly significant.

**Table 3:** Mean ± *SD* for color measurements of date powders

Variety	Treatment	L*	a*	b*
Rabi	OD	64.78 ± 0.73^e^	3.34 ± 0.22^d^	25.78 ± 0.75^d^
	SD	69.23 ± 0.98^d^	3.69 ± 0.22^c^	25.94 ± 0.75^d^
Aseel	OD	75.33 ± 0.31^b^	4.05 ± 0.57^ab^	30.49 ± 0.55^a^
	SD	77.14 ± 0.4^a^	3.91 ± 0.04^bc^	29.03 ± 0.26^b^
Dhakki	OD	72.68 ± 0.51^c^	4.18 ± 0.06^a^	27.88 ± 0.79^c^
	SD	71.83 ± 0.59^c^	4.24 ± 0.11^a^	26.71 ± 0.45^d^

Note

Means carrying different letters are significantly different (*p* < 0.05).

#### 3.4.2 Bulk density

Bulk density indicated packaging behavior of product that depends upon combined effect of some unified factors such as particle size, interparticle forces, and strength of contact points. The date powders exhibited the pronounced difference among varieties and negligible difference among the treatments. The calculated values for dhakki were same for the treatments, that is, 0.45 g/cm^3^, while bulk densities of oven‐dried and spray‐dried aseel were 0.49 ± 0.03 and 0.52 ± 0.03 g/cm^3^, respectively. Almost similar results were found for rabi. Sablani et al. (2008) prepared oven‐dried date powder with the bulk density ranged from 0.658 to 0.787 g/cm^3 ^(Figure 3). The variation was due to treatments where varying amounts of maltodextrin were used, whereas in current research, drying aid was constituted of gum Arabic and maltodextrin; therefore, results showed slightly lower bulk density, because higher bulk density was related to the higher concentrations of maltodextrin (higher polymers of glucose). While Acacia gum has lesser bulk density, this combination gave bulk density in the range of 0.45–0.52 g/cm^3^.

#### 3.4.3 Solubility

Solubility index of all the treatments and varieties indicated nonsignificant variations. The highest solubility for oven dried and spray dried was 83% followed by oven‐dried rabi and spray‐dried dhakki with values of 81.22% and 80.49%, respectively (Figure 2). Other treatments and varieties did also show same results. Food powders presented varying degree of solubility index because they can be supplemented along with water. Researchers found the solubility index of date powders in the range of 67%–88% depending upon carrier agents, conditions of preparations, and type of raw material (Manickavasagan et al., 2015; Sablani et al., 2008).

**Figure 2:** Means of solubility (%) and wettability time (s) of date powders

#### 3.4.4 Wettability time (s)

Wettability time varied among the varieties. The highest time was taken by spray‐dried dhakki with 126 ± 6.56 s followed by oven‐dried dhakki with 125 ± 5.57 s (Figure 2). The minimum time was taken by oven‐dried rabi with 60.67 ± 1.53 to 77 ± 4 s for spray‐dried rabi. Oven‐dried aseel powder took 110.33 ± 4.16 s, while spray dried took 101 ± 03 s. Similar results were revealed by Manickavasagan et al. (2015) for date powder where different carrier agents, maltodextrin and gum Arabic, were used, and the range of wettability time was 5.2–9.7 s for maltodextrin‐added powder while 145–169 s for gum Arabic‐added powder. Wettability of powders was affected by the ingredients; smaller molecules with higher water affinity took less time for wetting (Sablani et al., 2008).

#### 3.4.5 Hygroscopicity

Mean values for hygroscopicity showed minimal difference among treatments and varieties. And the hygroscopicity almost equal values only dhakki OD and SD showed little difference, that is, 0.06 g/gram of powder (Figure 3). Mean squares showed nonsignificant difference among all values. Manickavasagan et al. (2015) and Sablani et al. (2008) found range of hygroscopicity in date powders from 0.03 to 0.08 g/gram of powder and 4% to 6.2%, respectively. Hygroscopicity can vary from powder to powder depending upon the constituents of powders (Shishir, Taip, Aziz, & Talib, 2014).

**Figure 3:** Means for hygroscopicity and bulk density of date powders

#### 3.4.6 Glass transition temperatures

The stickiness of low molecular weight sugars was high due to their tendency of lower transition temperature, which was exceedingly related to higher moisture contents. The higher moisture contents resulted in lower glass transition temperatures. The glass transition temperature (*T*_g_) is the temperature at which physical state of the food material undergoes viscous flow mechanism and has higher moisture contents and storage temperature transforms the amorphous state of product to glassy material that ultimately converts into rubbery state which results into very low surface viscosity. Material with minimal viscosity starts to adhere to itself and becomes very sticky. Date particles have rubbery nature due to dominance of low molecular weight sugars; therefore, the likelihood of their stickiness was higher during short storage period. The glass transition temperature was increased by adding drying aid that ultimately improves the *T*_g_ of the powders. In the preparation of fruit powders, mango powder, tamarind powder, pineapple powder, and guava powder, mostly high molecular weight food polymers are used that complement the lower glass transition temperatures of the original product and increase its thermal stability (Jaya & Das, 2004; Shishir et al., 2014).

The results were also satisfactory in relation to *T*_g_. The free‐flowing powder with higher thermal stability was produced due to higher glass transition temperature compared to room temperature. The results revealed that drying method affected the moisture contents which ultimately affect the *T*_g_ of the powders. The initial, midpoint, and end point glass transition temperatures were calculated through differential scanning calorimeter, and the spray‐dried powders with less water activity showed higher thermal stabilities compared to the oven‐dried powders. The difference among varieties was not significant that accentuated the further effect of drying method. Table 4 shows that glass transition temperatures vary from 45.6 ± 1.34 to 48.6 ± 0.98°C within same variety with different drying method. Similar trend was prominent in other varieties where glass transition temperature is a function of water activity which varied with the drying methods.

**Table 4:** Glass transition temperature (°C) and water activity (aω) of the oven‐dried and spray‐dried powders

Glass transition temperature (°C)	Drying method	Rabi		Aseel		Dhakki	
		OD	SD	OD	SD	OD	SD
	W.A (aω)	0.20 ± 0.01	0.183 ± 0.1	0.199 ± 0.002	0.178 ± 0.001	0.193 ± 0.001	0.167 ± 0.001
*T*_gi_		45.6 ± 1.34	48.6 ± 0.98	44.3 ± 2.1	47.2 ± 1.72	45.3 ± 0.12	48.1 ± 0.89
*T*_gm_		48.9 ± 2.23	50.1 ± 1.21	47.6 ± 1.23	49.1 ± 1.1	47.9 ± 0.62	50.3 ± 0.97
*T*_ge_		52.3 ± 1.67	53.2 ± 1.31	49.9 ± 1.68	51.7 ± 0.93	50.9 ± 2.23	53.1 ± 1.31

Abbreviations: *T*_ge_, end point glass transition temperature; *T*_gi_, initial temperature; *T*_gm_, midpoint glass transition temperature. OD, Oven Dried; SD, Spray Dried.

## 4 CONCLUSION

Drying plays an important role in value addition for date processing. Spray drying is better method as water activity is lesser in spray‐dried date powder with minimal effect on nutritional profile as well as physicochemical properties, which results in more thermostable product with higher shelf life. DSC provides clearer picture that free‐flowing powder with no crystalline structure is produced; therefore, a stable nutraceutical date powder having higher shelf life can replace tabletop sugar.

## CONFLICT OF INTEREST

The authors declare that they have no conflict of interest.

## ETHICAL APPROVAL

This article does not contain any studies with human participants or animals performed by any of the authors. It is further certified that human and animal testing is unnecessary in this study.

## INFORMED CONSENT

For this type of study, formal consent is not required.
